# Progressive Collateral Stenosis Leading to Symptomatic Chronic Total Occlusion

**DOI:** 10.7759/cureus.12524

**Published:** 2021-01-06

**Authors:** Farhan A Shah, Andrew Maiolo

**Affiliations:** 1 Internal Medicine, LewisGale Medical Center, Salem, USA; 2 Cardiology, LewisGale Medical Center, Salem, USA

**Keywords:** cardiology, interventional cardiology, chronic total occlusion, angioplasty and stenting

## Abstract

We present a case of chronic total occlusion (CTO) in a functional 79-year-old female with no past history of coronary artery disease, who was previously asymptomatic due to robust collateral circulation. A 79-year-old Caucasian female presented to the emergency department complaining of chest pain radiating to the neck, jaw, left arm with associated numbness in the left fingers, that had started earlier in the day. She has no previous cardiac history and never had similar symptoms before. Troponin levels were negative. Nuclear stress test showed findings worrisome for ischemia and was a high-risk exam. The patient underwent diagnostic angiography. There was complete total occlusion of the mid right coronary artery, with collateral circulation supplying the distal right coronary artery territory. Ultimately, it found that progressive stenosis of the left anterior descending (LAD) artery led to inadequate collateral circulation and completely occluded the right coronary artery’s territory, causing the patient’s new-onset angina. Afterwards, the patient underwent percutaneous coronary intervention (PCI). Successful implantation of two drug-eluting stents occurred. The final angiographic result was 0% residual stenosis and Thrombolysis in Myocardial Infarction (TIMI)-3 flow. CTO affecting one or more coronary arteries is not uncommon in patients taken to the catheterization laboratory. However, despite recent advancements in PCI outcomes, treatment of CTO by PCI remains relatively low, due to fear of adverse outcomes such as cardiac perforations. Recent research has supported the safety of performing PCIs on patients with CTO. This case report further reinforces the need to approach treating CTO via angioplasty.

## Introduction

Coronary chronic total occlusion (CTO) is defined as Thrombolysis in Myocardial Infarction (TIMI)-0 flow for more than three months in a coronary artery [1]. Efficacy and risks of CTO percutaneous coronary intervention (PCI) have been under review. We present a case of CTO in a functional 79-year-old female with no past history of coronary artery disease, who was previously asymptomatic due to robust collateral circulation.

## Case presentation

The patient is a 79-year-old Caucasian female with a past medical history of chronic lymphocytic leukemia, hypertension, hyperlipidemia, type 2 diabetes mellitus, who presented to the emergency department complaining of sharp, intermittent chest pain that radiated to the neck, jaw, left arm with associated tingling and numbness in the left fingers. She never had these symptoms before. Initial and repeat troponin levels were negative. Physical exam revealed normal S1, S2, without any abnormal heart sounds heard, including no murmurs, gallops, or rubs, and had a normal rate and rhythm.

Chest X-ray showed stable cardiomegaly. Nuclear stress test showed findings worrisome for ischemia of the apical septal, anterior apical lateral and basal inferolateral wall, significant left ventricular dysfunction with abnormal wall motion, characterized as a high risk exam. Ejection fraction was 31% and global hypokinesis was present.

The patient underwent diagnostic catheter angiography. Left anterior descending (LAD) artery showed 80% stenosis (TIMI-3 flow) with collateral circulation supplying the distal right coronary artery territory. The left circumflex artery gave off minimal left-to-right collaterals, as well, filling the distal right coronary artery territory (Figure 1).

**Figure 1:** Left anterior descending artery showed 80% stenosis (yellow arrow) with collateral circulation supplying the distal right coronary artery territory (red arrows)

There was CTO of the mid right coronary artery (Figure 2). Ultimately, it was noted that the progressive stenosis of the LAD artery leading to its inadequate collateral circulation to the completely occluded right coronary artery’s territory, further worsened the ischemia and was most likely the cause of the patient’s new-onset angina.

**Figure 2:** Chronic total occlusion of right coronary artery (red arrow)

Afterwards, the patient underwent PCI. The guide wire could not pass through the mid right coronary artery due to CTO. However, the guide wire was able to cross through a micro channel into the distal vessel. Several attempts were necessary with varying sized balloons to predilate the artery. Successful implantation of two drug-eluting stents occurred (Figure 3). Final angiographic result was 0% residual stenosis and TIMI-3 flow. The patient was discharged the following day and further staged PCI of the mid LAD artery would occur in two-four weeks.

**Figure 3:** Guide wire crossed into the distal vessel (red arrow); successful implantation of drug-eluting stent (yellow arrow)

## Discussion

The definition of CTO is a complete obstruction of a coronary artery, with a TIMI 0 or TIMI 1 flow and the duration of the occlusion being greater than three months [1]. CTO is thought to be found in roughly 20% of all patients who are referred for coronary angiography. CTO prevalence in patients with known coronary artery disease has been documented as ranging from 30% to 50%. According to data in the National Heart, Lung, and Blood Institute Dynamic Registry between 1997 and 1999, in patients who underwent PCI, CTOs were frequent and more likely encountered in the older population. At least one CTO was present in 36.5% of patients < 65 years, 39.1% seen in those who were between 65-79 years, and 40.7% seen in those ≥ 80 years of age. Specifically, the right coronary artery was found to be the most commonly affected coronary vessel, followed by the LAD and left circumflex arteries [1].

Despite recent advancements in PCI outcomes, revascularization treatments of CTO by PCI historically remains low, due to fear of adverse outcomes such as cardiac perforations. PCI is only performed on around 10% to 15% of patients with CTO [1]. According to the Bypass Angioplasty Revascularization Investigation (BARI) trial, the presence of a CTO was the most prevalent angiographic factor leading to the decision against enrollment and subsequent referral for coronary artery bypass graft (CABG) and treatment with medical therapy. When a CTO was present in the BARI trial, 10% received PCI, 40% received CABG, while 50% received medical therapy. When a CTO was not present, instead 35% underwent PCI, 30% underwent CABG, and 35% received medical therapy [2,3]. In the past, PCI for a CTO had low success rates of about 50%, leading to the consideration that CABG was the gold standard of achieving complete revascularization [3]. Treating CTO by PCI is considered technically challenging, due to several difficulties such as the inability to cross the obstruction with a guidewire, the inability to cross the obstruction with a balloon following the successful guidewire passage, the inability to deliver or expand a stent across the lesion, or ultimately the perforation of the vessel with a guidewire [1]. However, recent research has supported the safety and efficacy of performing PCIs on patients with CTO, especially with novel PCI techniques.

The four main techniques for successful PCI of CTO, include antegrade wire escalation, antegrade dissection and reentry (ADR), retrograde wire escalation, and retrograde dissection and reentry [3]. As seen in the PROGRESS CTO registry (Prospective Global Registry for the Study of Chronic Total Occlusion Intervention), skilled operators can have high success rates of 91% with low major complication rates of around 1.7% [3]. This is further endorsed by the 2011 American College of Cardiology/American Heart Association guidelines for PCI which state: “PCI of a CTO in patients with appropriate clinical indications and suitable anatomy is reasonable when performed by operators with appropriate expertise” [4].

Fractional flow reserve (FFR) is a coronary catheterization technique used to determine if coronary artery stenosis is significant enough to justify PCI. It is defined as “the maximal blood flow to the myocardium in the presence of a stenosis in the supplying coronary artery, divided by the theoretical normal maximal flow in the same distribution” [5]. FFR has shown persistent ischemia in CTO lesions despite collaterals, indicating that the collateral circulation of CTOs are not sufficient to correct ischemia [3]. In a study comparing 50 CTO patients versus 50 patients in a non‐CTO control group, FFR of the ischemic zone post-PCI improved to the same absolute level in both CTO and non-CTO lesions, meaning efficacious PCI on CTO lesions resulted in an even greater relative benefit than their non-CTO counterparts, as evidenced by FFR improvement [1,6].

## Conclusions

Despite the technically challenging nature of CTO PCI, newer techniques and guidelines backing its efficacy have led to its increasing usage and subsequent shift in the clinical interventional management of patients with CTO.
